# Influence of chemical composition on the amount of second phases precipitates and transformation temperatures of TiNiPdCu shape memory alloys prepared through novel powder metallurgy route

This article has been retracted.

**DOI:** 10.1039/d3ra05513b

**Published:** 2023-10-09

**Authors:** Abid Hussain, Afzal Kan, Muhammad Imran Khan, Saif Ur Rehman

**Affiliations:** a Department of Mechanical Engineering, University of Engineering and Technology Peshawar Postcode 25120 Pakistan abidhussain@uetpeshawar.edu.pk; b Ghulam Ishaq Khan (GIK) Institute of Science, Engineering and Technology District Swabi Topi 23640 Khyber Pakhtonhwa Pakistan; c Institute of Industrial Control System Rawalpindi Pakistan

## Abstract

The chemical composition of TiNiPdCu high temperature shape memory alloys (HTSMAs) affects their microstructure and martensitic transformations. In TiNiPdC HTSMAs, second phase precipitates were found. Extremely high densities of nanoscale precipitates of TiPdCu and Ti_2_Pd of particle size 0.8–4.4 μm were found to be produced by the TiNiPdCu alloys. It was found that the TiPdCu-type precipitates were favoured by the preferential migration of Cu atoms towards the heterogeneous nucleation sites, which in turn favoured the fine Ti_2_Pd-type precipitates. Due primarily to their high-temperature stability, these precipitates significantly strengthened the resistance against transformation-induced plasticity and creep deformation, especially at high loads and high temperatures. High concentrations of these nanoscaled precipitates led to a significant rise in transformation temperatures by 12% and a small decrease in thermal hysteresis by 30%. It was anticipated that the current research findings will have a significant positive impact on the creation of HTSMAs that maintain their benefits of simplicity of manufacture. The HTSMAs developed in current research are beneficial for high temperature sensors and actuators at optimum cost.

## Abstract 2

The chemical composition of TiNiPdCu high temperature shape memory alloys (HTSMAs) affects their microstructure and martensitic transformations.

## Introduction

Alloys with higher martensitic transformation temperatures—at least greater than 100 °C—are known as HTSMAs. High temperature shape memory actuators have drawn a lot of attention in recent years, particularly for use in power production, automotive, and space exploration applications.^1–5^ HTSMAs have numerous potential applications in aerospace and aviation, such as high temperature solid state actuators, adaptive chevrons attached to aircraft core exhausts for noise reduction and fuel efficiency, variable area or variable geometry inlets, high force actuation systems, actuators for satellite deployment of space structures, deployable shields and protection screens, and seals for booster rinsing.^6–10^ HTSMAs have also been suggested for a variety of automotive applications, particularly for engine management and fuel control.^11^ HTSMA could also be used in energy exploration for downhole oil and gas applications such as flow safety valves, control valves, and tiny actuators.^12^ Another conceivable application for HTSMAs is in energy exploration for downhole oil and gas applications such as flow safety valves, control valves, and tiny actuators.^13^ Using HTSMA thin films, Orbital Research, Inc. has created a strain gauge for a pressure transducer that takes advantage of the superelastic features of HTSMAs.^14^ As these are only a few of the potential applications of HTSMAs, there are certainly many more that need to be researched. HTSMAs are still not commonly used in real-time commercial applications due to their poor cold workability and poor high temperature functional properties.^15^ High temperature applications are not acceptable for binary TiNi shape memory alloys.^16^ For the aforementioned applications, some ternary alloys based on TiNi, such as TiNiPt, TiNiAu, TiNiZr, TiNiPd, and TiNiHf, have demonstrated appropriate transition temperatures.^17–20^ Alloys made of TiNiPd, TiNiPt, and TiNiAu have a low hysteresis and a high temperature shape memory effect. A review paper by Ma *et al.* contains a thorough analysis of the aforementioned HTSMAs.^4^ By altering the concentration of ternary alloying components within the temperature range of 100–500 °C, the transformation temperatures in these alloys can be adjusted. These alloys' somewhat greater price in comparison to other HTSMAs is a drawback.^18,21^ Although the thermal hysteresis of the considerably less expensive TiNiHf and TiNiZr alloys is substantially larger than 45 K, they are not appropriate for actuator applications despite having high transformation temperatures. Additionally, the TiNiHf- and TiNiZr-based alloys both have extremely poor cold workability, making it nearly impossible to increase their high temperature stability using standard strengthening techniques like precipitation strengthening and strain hardening.^22–24^ In comparison to previous TiNi-based ternary HTSMAs systems, TiNiPd-based ternary HTSMAs offer an appealing combination of high transformation temperatures (TT), little hysteresis, good workability, and a relatively lower price.^25–29^ Like any other metallic material, creep deformation and transformation-induced plasticity significantly impair the functional performance of TiNiPd-based alloys at high temperatures.^30–32^ TiNiPdCu-based high temperature system has recently been proposed by research, specifically for high temperature shape memory effect (SME) applications. Due to a peculiar nanoscale precipitation behaviour, these alloys were discovered to display an outstanding behaviour in terms of their high temperature cyclic stability and creep properties, especially in difficult working conditions. Additionally, because of this particular precipitation behaviour involving lattice defects created during cold working, TiNiPd-based HTSMAs can now exploit the precipitation strengthening mechanism, which is ordinarily not allowed because of their hereditary poor cold workability.^32–34^ Numerous study reports have been published thus far on numerous significant elements of the TiNiPdCu alloy system. The goal of the ongoing research is to examine how chemical composition affects the temperatures of transition and the second phase precipitates. For actuator-type applications, small hysteresis is a crucial requirement. In current research work, HTSMAs with low hysteresis is developed, which is most suitable for high temperature sensors and actuators. The HTSMAs developed through novel powder metallurgy route are more economical as compared to Ar-arc melting method. The thermal hysteresis in current research work is reduced to 19 °C which is a big achievement in this research work. The minimum research work obtained in previous research work is 23 °C.

## Experimental section

### Materials and methods

Powders of titanium (Ti), nickel (Ni), copper (Cu), and palladium (Pd) were used to create alloys. The Ti, Ni, and Cu powders came from FS Corporation in Lahore, Pakistan, with a purity of 99.1%, while the Pd powders came from YURUI (SHANGHAI) Chemical Co., Limited in China with a purity of more than 99%, as shown in Table 1. The evaluation of the powder's particle sizes using Image-J software produced values for Ti, Ni, Cu, and Pd of 35 m, 2 m, 2.5 m, and 51 m, respectively. Applying the conversion formula, which converts atomic percentage into weight percentage and accounts for up to four decimal places in grams allowed for the accurate measurement of element masses.

**Table 1:** Powder purity (%) and particle size (μm)

Metal (powder)	Purity (wt%)	Particle size (μm)
Ti	99.3	35
Ni	99.3	2
Cu	99.3	2.5
Pd	99.1	51

### Mixing of Ti, Ni, Pd and Cu powders

The measured elements were cleaned for five minutes in an ultrasonic cleaner using methanol (CH_3_OH), and then they were combined according to the prescribed compositions. The materials were cold-compacted at an 800 MPa pressure after the blending procedure.

### Sintering of compacted powders in vacuum furnace

The compressed compositions underwent sintering at 950 °C in a vacuum furnace with an argon (Ar) environment to prevent oxidation. To achieve the correct composition and avoid the development of oxides or nitrides, the furnace chamber had to be properly evacuated of air (oxygen) before 99.99% pure argon gas was introduced. The alloys were created using a non-consumable DC electric arc melting furnace, producing 5 gram buttons. A copper crucible that had been water-cooled and a tungsten electrode were used in the melting process. To thoroughly clean the copper crucible and remove any surface impurities, paper and acetone were used for grinding. The furnace chamber was repeatedly evacuated to 1 × 10^−2^ mbar after being initially purified with 99.98% pure argon gas in order to remove oxygen. The chamber was evacuated to 1 × 10^−4^ mbar by repeating this procedure. In order to aid the creation of an electric arc between the tungsten electrode and the copper crucible, a small amount of argon gas was then added. The establishment of the proper medium for the arc formation required the presence of this argon.

Seven alloys with various copper (Cu) contents were produced using this method (Ti_50_Ni_25_Pd_25_, Ti_50_Ni_22_Pd_25_Cu_3_, Ti_50_Ni_21_Pd_25_Cu_4_, Ti_50_Ni_20_Pd_25_Cu_5_, Ti_50_Ni_19_Pd_25_Cu_6_, Ti_50_Ni_17.5_Pd_25_Cu_7.5_, and Ti_50_Ni_15_Pd_25_Cu_10_); they were given the names 0Cu, 3Cu, 4Cu, 5Cu, 6Cu, 7.5Cu, and 10Cu to reflect the atomic percent compositions of copper in each alloy.

### Homogenization

A homogenization method is necessary to establish a consistent chemical composition across the volume of the generated alloys. Each alloy button was put within a quartz tube that was vacuumed to a pressure of 1 × 10^−3^ mbar using rotary and diffusion pumps. The quartz tube was then sealed and completely filled with pure argon gas. The sealed quartz tubes with the alloy buttons were added after the tube furnace had been heated to 950 °C. The alloy buttons were loaded at a high temperature in order to avoid any potential precipitation during gradual heating. The alloy buttons were quickly quenched in ice water after spending two hours at 950 °C to avoid the formation of precipitates during the slow cooling process. The alloy buttons' structural integrity and prevention of oxidation require the use of quartz tubes during the quenching process.

### Solution treatment

Individual samples were placed within distinct quartz tubes after being evacuated, and then the solution treatment procedure was started by filling the tubes with pure argon gas. The samples were then put into a tube furnace that had been warmed to 900 °C. For two hours, the samples were kept at 900 °C inside the tube furnace. After this procedure, the samples were quickly cooled while still being contained inside quartz tubes. To avoid the tubes breaking, this chilling operation was carried out in cold water.

### Annealing

The samples were annealed at 950 °C after the solution treatment in order to evaluate their properties under this circumstance and compare them to their characteristics after the solution treatment. The samples from the alloys made up of 0Cu, 3Cu, 4Cu, 5Cu, 6Cu, 7.5Cu, and 10Cu were once more put inside quartz tubes after following the same steps as for the solution treatment. Then, a tube furnace that had been warmed to the necessary annealing temperature of 950 °C was filled with these sealed tubes. All seven alloys underwent annealing at this temperature. Following the predetermined soaking time, the samples were cooled within the furnace while still being contained inside the quartz tubes. Direct exposure to air and water was carefully avoided in order to protect the annealed characteristics and prevent any unexpected reactions.

### Aging

The remaining solution-treated samples underwent annealing at 700 °C to examine the characteristics of the aged samples and establish a comparison with their counterparts. Samples from the 0Cu, 3Cu, 4Cu, 5Cu, 6Cu, 7.5Cu, and 10Cu alloys were inserted within quartz tubes using a similar approach to that used for the solution-treated samples. These sealed tubes were put into a tube furnace after it was preheated to the 700 °C aging temperature. Then, all seven alloys underwent a six-hour maturation period at this temperature. The samples were quenched in water while remaining inside the quartz tubes once the soaking period was finished. As a result, the quartz tubes were not harmed during the aging process. This method made it easier to preserve the old buildings without any unfavourable interactions with air or water.

### Scan electron microscopy (SEM)

The materials were mechanically ground before going through scanning electron microscopy (SEM). With the aid of an exacting fine polishing procedure, alumina slurry with 0.5 micron-sized particles was used. The materials were appropriately prepped before being put into the SEM for examination.

### X-ray diffractometry (XRD)

In order to collect XRD patterns for this work, a computer-controlled X-ray diffractometer model JDX-99C from JEOL Japan was used. The diffractometer used Cu Kα radiation (=1.5406) operating at voltage of 40 kV and current of 20 mA at ambient temperature. Between 20° and 80°, incidence angle 2 was noticed. The detected XRD patterns were matched to the widely utilised Powder Diffraction File (PDF) in the International Centre for Diffraction Data (ICDD) database in order to interpret the findings. This comparison was done to determine the atomic makeup of the various phases that were present in the samples. This identification was made by comparing the intensity of the diffracted peaks with matching diffraction angles' *d*-spacing.

### Differential scanning calorimetry (DSC)

DSC is a widely used method for precisely determining a specimen's thermal characteristics. The heat transferred from the samples during procedures like heating, cooling, or isothermal holding is directly measured by this differential approach. DSC can look at different thermal events occurring inside the samples by tracking the amount of energy needed to maintain a certain temperature. A phase transition in the sample causes an abrupt change in heat release or absorption during heating or cooling. The DSC graph shows these transitions as discrete peaks. These peaks offer important information about the transitions that are taking place in the sample.

## Results and discussions

### Microstructural analysis of solution treated TiNiPdCu shape memory alloys (SMAs) with varied Cu content

Images taken using a SEM that show the microstructure of the 0Cu, 3Cu, 4Cu, 5Cu, 6Cu, 7.5Cu, and 10Cu alloys after solution treatment are shown in Fig. 1a–g. Discrete second-phase precipitates with low density can be seen randomly positioned along the grain boundaries of all seven alloys. Across the array of seven alloys, these precipitates have an average size between 0.8 and 4.4 μm using image J and Figi software and consistently display a nearly uniform round or elliptical shape. Notably, the addition of Cu had no effect on how big these precipitates were.

**Fig. 1:** SEM images of second phase precipitates generated in solution-treated samples of (a) 0Cu, (b) 3Cu, (c) 4Cu, (d) 5Cu, (e) 6Cu, (f) 7.5Cu and (g) 10Cu SMAs.

Energy-dispersive X-ray spectroscopy (EDS) analysis was carried out to confirm the chemical composition of the original elements and second-phase precipitates. Fig. 2 displays the EDS spectra, and Table 2 lists the associated chemical compositions. According to the information in Table 2, the second-phase precipitates that develop at the grain boundaries for the other six alloys and the 0Cu alloy are both composed of Ti_2_Ni(Pd) and Ti_2_Ni(Pd, Cu). These forms of precipitate are frequently found in NiTi-based alloys that are high in titanium (Ti).^33^ Due to their lower melting point compared to the matrix, second-phase precipitates of Ti_2_Ni(Pd) were seen during the solidification process.^35^ Equivalent kinds of precipitates were seen to occur in ternary TiNiPd alloys when Pd concentrations are above 10%, according to research. These discoveries led researchers to conclude that the addition of copper has no effect on the underlying microstructure of quaternary alloys. As seen when Scandium (Sc) in the form of Sc_2_O_3_ is added to TiNiPd, the injected copper remains within the solid solution matrix and does not cause any additional secondary phase precipitation.^26,36^ Suzuki *et al.* also observed the production of second-phase precipitates containing TiB_2_ when 0.2% Boron (B) was added to Ti_50_Pd_30_Ni_20_ in place of Ni.^37^

**Fig. 2:** EDS spectrums shown for solution treated samples of 0Cu, 3Cu, 4Cu, 5Cu, 6Cu, 7.5Cu and 10Cu alloys.

**Table 2:** EDS spectrums shown for solution treated samples of 0Cu, 3Cu, 4Cu, 5Cu, 6Cu, 7.5Cu and 10Cu alloys

Alloy name	Analysis region	Ti (%)	Ni (%)	Pd (%)	Cu (%)
0Cu	Overall alloy	49.63	23.46	26.91	
	Ti_2_Ni	56.4	26.7	16.9	
3Cu	Overall alloy	50.14	22.73	24.47	2.66
	Ti_2_Ni	55.4	25.8	14.7	4.1
4Cu	Overall alloy	48.87	23.51	23.40	4.22
	Ti_2_Ni	57.6	21.5	13.3	7.6
5Cu	Overall alloy	49.54	24.37	20.97	5.12
	Ti_2_Ni	61.3	20.7	14.1	3.9
6Cu	Overall alloy	48.77	17.07	27.42	6.74
	Ti_2_Ni	60.4	18.3	13.8	7.5
7.5Cu	Overall alloy	51.08	14.39	27.72	6.82
	Ti_2_Ni	64.8	19.2	14.3	1.7
10Cu	Overall alloy	50.87	14.30	24.68	10.16
	Ti_2_Ni	66.7	16.9	11.8	4.6

### Effect of aging temperature on microstructure of TiNiPdCu alloys with varied Cu content

The samples were subjected to SEM analysis to look into the effects of various aging temperatures on the SMAs. SEM pictures of the 0Cu alloy aged at 400, 500, 600, and 700 °C are shown in Fig. 3. Only the second-phase precipitates, which were first generated during the solidification process, are visible in these SEM images. SEM images of the 5Cu alloy under the same aging circumstances are shown in Fig. 4a–d. The second-phase precipitates located along the grain boundaries are visible in these images, confirming their presence. Fig. 4a demonstrates that at an aging temperature of 400 °C, the precipitation process had not begun. When the aging temperature was raised to 500 °C, exceptionally fine precipitates with a luminous appearance were seen. As the aging temperature was elevated to 600 °C, precipitation density increased. As the aging temperature rose to 700 °C, the size of the precipitates grew larger. Both the areas along the grain borders and the core of the grains contained these precipitates.

**Fig. 3:** SEM images of the microstructure and grain boundaries in 0Cu alloys after 6 hours of ageing at (a) 400 °C, (b) 500 °C, (c) 600 °C, and (d) 700 °C.

**Fig. 4:** SEM images presenting the microstructure and grain boundaries in 5Cu alloys after 6 hours of aging at temperature of (a) 400 °C, (b) 500 °C, (c) 600 °C and (d) 700 °C.

Fig. 5a–d SEM images show the precipitation patterns of 7.5Cu alloys that underwent the same aging conditions. The sample was aged at 400 °C, and Fig. 5a shows the sample's microstructure. It demonstrates how the precipitation process began with the production of incredibly fine precipitates along the grain boundaries. Notably, the absence of precipitation within the grain core confirms the function of the grain borders as nucleation sites. Fig. 5b depicts the microstructure of an alloy aged at 500 °C, which has two types of precipitates scattered on both sides of the grain boundaries. These precipitates are larger than those created at 400 °C. Fig. 5c demonstrates that as the aging temperature increases to 600 °C, so the precipitate density rises. Both types of precipitates arise heterogeneously at this temperature along grain borders and within the grain interior. These precipitates, which are seen in Fig. 5b and c, have varying-length thread-like architectures. The microstructure of the SMAs aged at 700 °C is shown in Fig. 5d, and it is clear that low-density precipitates with comparatively bigger sizes have formed. When an alloy is aged at 700 °C, its precipitation behaviour dramatically changes from that seen at 500 °C and 600 °C. It's interesting to note that Khan *et al.* also observed the annealing-induced development of nanoscale precipitates in the same alloy after annealing at 823 K, 873 K, and 923 K for 60 minutes after 40% cold deformation.^34^ Although they differed from the precipitates produced in the current experiment, the precipitates detected in the annealing process showed nanoscale dimensions (100–300 nm) and a variety of morphologies (including elliptical and rod-like shapes). Furthermore, the precipitation behaviour observed during the annealing phase was markedly different from that observed during the aging process. In the scenario involving cold deformation followed by annealing, deformation-induced defects resulted in the establishment of heterogeneous nucleation sites. In the context of age hardening, the commencement of the precipitation process was connected to high-energy grain boundaries acting as nucleation sites.^38^

**Fig. 5:** SEM images presenting the microstructure and grain boundaries in 7.5Cu alloys after 6 hours of aging at temperature of (a) 400 °C, (b) 500 °C, (c) 600 °C and (d) 700 °C.

SEM images of aged 10Cu alloys are shown in Fig. 6a–d. Fig. 6a shows the sample's microstructure after being aged at 400 °C and demonstrates how extremely fine precipitates started to form on both sides of the grain boundaries. However, as shown in Fig. 5a, these precipitates were greater in size than the 6Cu alloy sample that had been aged at 400 °C. The microstructure of the SMAs aged at 500 °C are shown in Fig. 6b, where the two types of precipitates are greater than those that occurred in the same alloy at 400 °C. Fig. 6c shows that the density of the precipitates increases when the aging temperature is raised to 600 °C. Ti_2_Pd and TiPdCu precipitates are observed to be heterogeneously generated at this temperature both along the grain borders and inside the grain. Fig. 6b and c show the structure of the precipitates as thread-like structures of various lengths. The microstructure of the SMAs aged at 700 °C are depicted in Fig. 6d, emphasising the formation of precipitates with low density and large size. When the SMAs were aged at 700 °C, its precipitation behaviour notably differed from that seen at aging temperatures at 500 °C and 600 °C.

**Fig. 6:** SEM images presenting the microstructure and grain boundaries in 10Cu alloys after 6 hours of aging at temperature of (a) 400 °C, (b) 500 °C, (c) 600 °C and (d) 700 °C.

It is known that a precipitate with a stronger contrast in SEM images denotes the presence of heavier elements, specifically those with higher atomic numbers. A precipitate with a darker contrast, on the other hand, denotes the existence of lighter elements, or atoms with lower atomic numbers.^39^ As can be seen from the periodic table, Ti is lighter than the other constituent elements since it has a lower atomic number than Ni, Pd, and Cu. As a result, the presence of Ti-rich and Ti-lean precipitates are denoted, respectively, by darker and brighter contrasts.^39^ EDS analysis was carried out to determine the specific composition of the freshly generated precipitates as a result of aging at various temperatures, and the results were summarised in Table 3. The darker and brighter contrast particles in Fig. 5 and 6 are Ti_2_Pd (Ti-rich) and TiPdCu (Ti-lean) precipitates, respectively, according to the EDS analysis and the SEM images. In both forms of precipitates, it can also be seen that the Ni content is lower than the desired composition. This suggests that the precipitates' production increased the matrix's Ni content while lowering its Ti concentration.

**Table 3:** EDS spectrums shown for aged samples of 0Cu, 3Cu, 4Cu, 5Cu, 6Cu, 7.5Cu and 10Cu alloys

Alloy name	Analysis region	Ti (%)	Ni (%)	Pd (%)	Cu (%)
0Cu	Black precipitates	60.1	11.3	22.5	6.1
	White precipitates	37.5	10.6	26.3	25.6
3Cu	Black precipitates	57.8	11.4	23.7	7.1
	White precipitates	40.3	10.9	27.7	21.1
4Cu	Black precipitates	61.6	11.2	23.5	3.7
	White precipitates	40.1	10.9	27.6	21.4
5Cu	Black precipitates	56.9	12.2	25.6	5.3
	White precipitates	38.5	9.8	29.2	22.5
6Cu	Black precipitates	61.3	11.2	22.7	4.8
	White precipitates	37.7	12.3	27.6	22.4
7.5Cu	Black precipitates	59.5	12.1	23.3	5.1
	White precipitates	36.9	12.6	27.9	22.6
10Cu	Black precipitates	58.7	10.1	24.3	6.9
	White precipitates	39.7	11.2	28.9	20.2

When stoichiometric TiNiPd alloys (with a composition of Ti : Ni + Pd = 50% : 50%) are compared to the precipitation behaviour of 0Cu, 5Cu, 7.5Cu, and 10Cu alloys, it becomes clear that there was no precipitation process during the aging temperature range of 400 °C to 700 °C. The precipitation behaviour of 5Cu alloys is generally comparable to that of 0Cu alloy. At aging temperatures of 500 °C, 600 °C, and 700 °C, however, very fine precipitates with a greater contrast were seen, as shown in Fig. 4b–d. The precipitation behaviour of stoichiometric TiNiPd alloys changed significantly when 6% and 10% Cu were substituted for Ni. Precipitation started in both alloys along the grain boundaries at lower aging temperatures. The precipitates grew in size and density as the temperature rose, reaching their maximum at a temperature of 600 °C. However, the precipitates' size continued to increase while their density continued to decline at an aging temperature of 700 °C. Additionally, it was discovered that, at the same temperatures, the precipitates generated in the 10Cu alloys were greater than those in the 7.5Cu alloys.

### Effect of annealing temperature on microstructure of TiNiPdCu alloys with varied Cu content

The SEM microstructures of the 10Cu alloy after annealing at 450 °C, 550 °C, 650 °C, 750 °C, 850 °C, and 950 °C are shown in Fig. 7a–f. The relevant photographs are magnified more than usual in the insets. The precipitation behaviour of the annealed 10Cu alloy was unexpected. The microstructure of the 10Cu alloy after 450 °C annealing is shown in Fig. 7a. Notably, this sample's SEM image does not show any signs of precipitation, indicating that precipitation did not start at this annealing temperature. Fig. 7b presents the microstructure of the 10Cu alloy after it was annealed at 550 °C. Again, due to the fine and tiny size of the precipitates, the SEM picture in Fig. 7b does not show any visible precipitates.

**Fig. 7:** SEM images of 10Cu alloy annealed at (a) 450 °C, (b) 550 °C, (c) 650 °C, (d) 750 °C, (e) 850 °C and (f) 950 °C for 1 h.

In the sample that was annealed at 650 °C, a surprisingly dense population of fine precipitates was found, as shown in Fig. 7c. Fig. 7d and e illustrate how the precipitates' size was seen to have become larger and how their density seemed to gradually decrease after being annealed at 750 °C and 850 °C. In these samples, two separate precipitate types were visible, one with a brighter contrast and the other with a darker contrast. In SEM images, a precipitate with a higher contrast indicates the presence of heavier elements (with a higher atomic number), whereas a precipitate with a lower contrast indicates the presence of lighter elements (with a lower atomic number).^40^ It is commonly known that Ti is lighter than Cu, Pd and Ni.

### Phase analysis of solution treated TiNiPdCu SMAs with varied Cu content

Utilising an X-ray diffractometer with Cu Kα radiation (=1.5406), X-ray phase analysis was carried out. The martensite phase, specifically in the range of 20 to 80° at room temperature, was used to capture the XRD patterns. The main peaks were primarily found in the diffraction angle region of 30 to 60°, according to the XRD study. The XRD patterns of solution-treated TiNiPdCu alloys for the 0Cu and 3Cu compositions are shown in Fig. 8a and b. The B19 orthorhombic martensite phase's peaks are clearly visible in the XRD profile. This finding suggests that the alloys are made entirely of the B19 martensite phase at normal temperature. Notably, the XRD patterns cannot easily identify the secondary phase particles, such as Ti_2_Ni(Pd) in the 0Cu alloy and Ti_2_Ni(Pd, Cu) in the treated alloys, which are apparent in the SEM images shown in Fig. 1. Due to their small volume percentage, the treated alloys did not exhibit noticeable peaks for Ti_2_Ni(Pd) and Ti_2_Ni(Pd, Cu). The B19 martensite peaks consistently migrate towards lower 2 angles in TiNiPd alloys that contain Cu. The significant B19 (111) martensite peak that was first shown in Fig. 7b at an angle of 43° for the 0Cu alloy gradually shifts to lower angles for the next six alloys. The expansion of lattice constants is probably to blame for the change in diffraction angle observed with increased Cu concentration. This expansion is related to the introduction of Cu, whose atomic radius is greater than that of Ni (0.125 nm) Cu (0.128 nm).

**Fig. 8:** (a) XRD results of sintered and homogenized samples at 25 °C (0Cu, 3Cu, 4Cu, 5Cu, 6Cu, 7.5Cu, 10Cu), (b) XRD results of sintered, homogenized, and solution treated samples at 25 °C (0Cu, 3Cu, 4Cu, 5Cu, 6Cu, 7.5Cu, 10Cu), (c) XRD results obtained of, homogenized, solution treated and annealed samples at 25 °C (0Cu, 3Cu, 4Cu, 5Cu, 6Cu, 7.5Cu, 10Cu) and (d) XRD results of sintered, homogenized, solution treated and aged samples at 25 °C (0Cu, 3Cu, 4Cu, 5Cu, 6Cu, 7.5Cu, 10Cu).

### Phase analysis of TiNiPdCu SMAs aged at 700 °C with varied Cu content

For samples that underwent solution treatment and were then aged at 700 °C across seven distinct alloy compositions, the XRD patterns obtained at ambient temperature are shown in Fig. 8d. These patterns can be analysed to identify the B19 martensite phase, which is represented by four separate peaks: (002), (020), (111), and (022). However, there are discernible peaks in the 7.5Cu and 10Cu alloys that correlate to both the black and white precipitates.

Extremely fine precipitates emerge when alloys containing 0Cu, 3Cu, 4Cu, 5Cu, and 6Cu are aged at 700 °C. These precipitates are still undetectable in the XRD patterns, though. This behaviour can be due to these precipitates' small volume fractions, which make it impossible to discriminate between them using XRD analysis. Contrarily, when the 7.5Cu and 10Cu alloys are aged at 700 °C, visible peaks connected to the black and white precipitates are produced. The existence of different peaks suggests that secondary phase precipitates with a greater volume fraction are present. This result is consistent with the compositional information in Table 4 and the relevant ref. 41. Verification was successful, establishing that the peaks near the martensite reflection peaks on the left and right sides, respectively, correspond to Ti_2_Pd and TiPdCu. The XRD analysis results for precipitation tendencies were in perfect agreement with the microstructures shown in Fig. 3d, 4d, 5d, and 6d.

**Table 4:** Texture coefficient, particle size and lattice parameters

Alloys	TC			Particle size (μm)	Lattice parameters		
	002	020	111	4.4	*a* (nm)	*b* (nm)	*c* (nm)
Ti_50_Ni_25_Pd_25_	1.154	0.931	0.391	3.9	0.2681	0.4297	0.4599
Ti_50_Ni_22_Pd_25_Cu_3_	1.388	0.832	0.382	3.2	0.2698	0.4301	0.4613
Ti_50_Ni_21_Pd_25_Cu_4_	1.556	0.784	0.364	2.7	0.2739	0.4311	0.4625
Ti_50_Ni_20_Pd_25_Cu_5_	1.872	0.712	0.351	2.1	0.2792	0.4319	0.4638
Ti_50_Ni_19_Pd_25_Cu_6_	2.012	0.632	0.342	1.8	0.2794	0.4356	0.4652
Ti_50_Ni_17.5_Pd_25_Cu_7.5_	2.472	0.589	0.322	1.4	0.2796	0.4376	0.4661
Ti_50_Ni_15_Pd_25_Cu_10_	2.626	0.412	0.285	1.1	0.2799	0.4401	0.4671

### Phase analysis of TiNiPdCu SMAs annealed at 950 °C with varied Cu content

Fig. 8c shows the XRD profiles for the solution-treated and annealed samples of the 0Cu, 3Cu, 4Cu, 5Cu, 6Cu, 7.5Cu, and 10Cu alloys that were prepared at room temperature. In the 0Cu, 3Cu, 5Cu, and 6Cu alloys, the XRD profiles show the existence of four peaks indicated as (002), (020), (111), and (022), which correspond to the B19 martensite phase. The very fine precipitates generated after annealing in the 0Cu, 3Cu, 4Cu, 5Cu, and 6Cu alloys are not, however, visible in the XRD profiles. This anomaly can be attributable to these precipitates' low volume fraction, which makes them invisible to XRD examination. In the case of the 7.5Cu and 10Cu alloys, however, new peaks develop on the left and right sides of the 39.75° angle.

### Texture coefficient calculations and particle size

The three peaks displayed in Fig. 8a–d are orthorhombic B19, designated as B19 (002), B19 (020), and B19 (111). With the addition of Cu content, a consistent shift in B19 martensite peaks was observed, indicating that the Cu addition caused a change in the B19 martensite lattice constants. The orthorhombic B19 martensite lattice constants measured from the same XRD patterns are shown in Table 4. With the increase of Cu concentration, the lattice constants (*a*, *b*, and *c*) increased. Cu has a larger atomic radius (0.128 nm) than Ni (0.125 nm), which explains the rise in lattice constants.

The texture coefficient (TC) of a specific plane (*hkl*) is determined using the eqn (1).^42^1where *I*_r_(*hkl*) is the ratio of a plane's measured relative intensity (*hkl*) to its standard intensity obtained from the JCPDS data, *N* is the reflection number and *n* is the number of diffraction peaks. The three typical peaks ((002), (020), and (111)) have their TCs values calculated and reported in Table 4. The texture coefficient of the (002) peak (TC (002)) diminishes with increasing crystalline size, according to the results. The other structural characteristic of alloys (texture coefficient) is similarly illustrated in Table 4 as a function of crystalline size. The higher the value of TC (002) (>1), the more oriented along the *C*-axis.

### Effect of Cu addition on transformation temperatures for solution treated TiNiPdCu SMAs

It is clear from Fig. 9a that it is impossible to ascertain the transition temperature for sintered and homogenised alloys. Fig. 9b shows the DSC heating and cooling cycles of alloys with various Cu percentages (0Cu, 3Cu, 4Cu, 5Cu, 6Cu, 7.5Cu, and 10Cu), which were all subjected to a solution treatment at 900 °C for one hour. Plotted in Fig. 10 are the phase transition temperatures obtained from the DSC cycles in Fig. 9b. This comparative analysis sought to determine how the addition of various amounts of Cu (3%, 4%, 5%, 6%, 7.5%, and 10%) to the base 0Cu alloy affected the transformation temperatures. All alloys showed the same general trend, which showed a one-step martensite transition with precisely estimated peaks for the transformation temperatures. DSC curves are used to calculate transformation temperatures such as martensite start temperature (*M*_s_), martensite finished temperature (*M*_f_), austenite start temperature (*A*_s_), and austenite finished temperature (*A*_f_).

**Fig. 9:** DSC curves for 0Cu, 3Cu, 4Cu, 5Cu, 6Cu, 7.5Cu and 10Cu (a) homogenized alloys, (b) solution treated alloys (c) annealed alloys and (d) aged alloys.

**Fig. 10:** Effect of Cu addition on transformation temperature for solution treated alloys.

The *M*_s_ of the 0Cu alloy increased noticeably by 5 °C, moving from 143 °C to 148 °C, when 3% Cu was substituted for Ni. As a result, the austenite finish temperature (*A*_f_) increased by 6 °C, rising from 168 °C to 172 °C. In addition, the thermal hysteresis showed a small decrease of 1 °C, going from 25 °C to 24 °C. These empirical findings highlight the effect of substituting 3% Cu for Ni, which causes a significant increase in transformation temperatures and a slight decrease in thermal hysteresis. Similar to this, the *M*_s_ temperature of the 5Cu alloy increased further and was 10 °C higher than those of the 0Cu alloy as a reference, from 143 °C to 153 °C, and its *A*_f_ temperature increased by 8 °C, going from 168 °C to 176 °C. In addition, it was noted that the thermal hysteresis dropped from 25 °C to 23 °C by 2 °C.

Parallel to this, the transformation temperatures of the 7.5Cu alloy increased further and went up by 16 °C above the baseline 0Cu alloy. The *M*_s_ temperature of the 0Cu alloy specifically increased by 12 °C, rising from 143 °C to 155 °C. The *A*_f_ temperature increased simultaneously by 10 °C, rising to 178 °C from 168 °C. Additionally, it was noted that thermal hysteresis decreased by 2 °C, from 25 °C to 23 °C. These empirical results clearly show that adding 7.5% Cu to Ni led to a significant increase in TTs and a minor decrease in thermal hysteresis. The TTs of the resulting 10Cu alloy significantly increased when 10% of the Ni in the original 0Cu alloy was replaced with Cu. The *M*_s_ temperature increased by 36 °C, rising from 143 °C to 179 °C. The *A*_f_ temperature also increased noticeably by 50 °C, going from 168 °C to 218 °C. Notably, the thermal hysteresis dropped from 25 °C to 24 °C by 1 °C. It has been conclusively proven, based on the aforementioned experimental findings, that 10% Cu in place of Ni resulted in a large increase in transformation temperatures and a significant decrease in thermal hysteresis which is suitable for high temperature sensors and actuators.

There is no doubt that variations in the Ni/Pd mix are related to variations in transformation temperatures and heat. The results of research by Mercier *et al.* have demonstrated that the Cu concentration has no effect on the transition temperatures.^43^ T. Suburi.^38^ A shift towards higher transition temperatures can be attained by raising the Pd content and lowering the Ni concentration, as shown in the pseudo-binary phase diagram of TiNi–TiPd. The change in the Ni/Pd ratio is what caused this. The transition temperatures increase when the Ni content drops while the Pd content stays the same. As a result, there is an increase in the temperatures that are absorbed and released during the forward and reverse martensitic transformations. The Clausius–Clapeyron equation, which establishes a direct association between the elevation in transformation temperature and the accompanying rise in transformation heat, is also applied to support this occurrence.

### Effect of Cu addition on transformation temperatures for aged TiNiPdCu SMAs at 700 °C

Seven alloys that underwent a 700 °C aging process were the subject of a study to look at how aging affects phase transformation temperatures. Fig. 9d shows the DSC heating and cooling cycles for the alloys containing 0 Cu, 3 Cu, 5 Cu, 7.5 Cu, and 10 Cu. These alloys were first given a solution treatment before being aged at 700 °C. Fig. 11 reanalysis of the phase transformation temperatures derived from the DSC cycles in Fig. 9d allowed for a thorough comparison of how the addition of Ni with 3%, 5%, 7.5%, and 10% Cu affected the temperatures relative to the 0Cu alloy.

**Fig. 11:** Effect of Cu addition on transformation temperature for aged alloys.

A startlingly comparable pattern appeared in all the alloys, demonstrating a consistent one-stage martensite transition characterised by sharp peaks and accurately calculated transformation temperatures. The area under the cooling curve, which measures the transformation heat (*H*_c_) released during the forward transformation cycle, and the area under the heating curve, which measures the transformation heat (*H*_h_) absorbed during the reverse transformation cycle, both showed an increase in direct correlation with higher Cu content in the alloy.

In particular, the 0Cu alloy's *M*_s_ temperature increased by 8 °C, ranging from 142 °C to 150 °C. In addition, the temperature in the *A*_f_ increased by 7 °C, from 165 °C to 172 °C. Additionally, a 1 °C decrease in thermal hysteresis was noted, moving from 26 °C to 25 °C, as seen in Fig. 10. These experimental results led to the conclusion that the addition of 3% Cu instead of Ni significantly reduced transformation temperatures while just slightly increasing thermal hysteresis.

The *M*_s_ temperatures of the 5Cu alloy also increased by 11 °C, moving from 142 °C to 153 °C, but the *A*_f_ temperature increased by 10 °C, from 165 °C to 175 °C. Thermal hysteresis was also seen to drop by 1 °C, moving from 26 °C to 25 °C. Based on these experimental results, it was determined that substituting 5% Cu for Ni caused an increase in transformation temperatures and a modest drop in thermal hysteresis.

The 0Cu alloy's *M*_s_ temperature increased by 15 °C, going from 142 °C to 157 °C, while the *A*_f_ temperature increased by 13 °C from 165 °C to 178 °C. Based on these experimental findings, it was deduced that 7.5% Cu was substituted for Ni led to a significant increase in transformation temperatures and a modest drop in thermal hysteresis.

The transformation temperatures of the resulting 10Cu alloy increased noticeably when 10% Cu was added in place of Ni in the 0Cu alloy. The 0Cu alloy's *M*_s_ temperature climbed by 49 °C, from 142 °C to 191 °C, and its *A*_f_ temperature climbed by 43 °C, from 165 °C to 208 °C. The thermal hysteresis remains constant at 26 °C.

### Effect of Cu addition on transformation temperature annealed at 950 °C

The DSC heating and cooling cycles of the alloys 0Cu, 3Cu, 5Cu, 7.5Cu, and 10Cu are shown in Fig. 9c. These alloys were subjected to solution treatment and annealing at 950 °C. In order to compare how the phase transformation temperatures changed when Ni was substituted with 3%, 5%, 7.5%, and 10% Cu, in contrast to the 0Cu alloy, the phase transformation temperatures obtained from the DSC cycles in Fig. 9c were then re-plotted in Fig. 12. A single-stage martensite transition was found to be the defining characteristic of the highly uniform behaviour seen across all alloys. The well-defined peaks with exactly calculated transition temperatures can be seen in the DSC profiles. However, higher Cu contents in the alloy were correlated with higher transformation heat (*H*_c_) released during the forward transformation cycle (area under the cooling curve) and transformation heat (*H*_h_) absorbed during the reverse transformation cycle (area under the heating curve).

**Fig. 12:** Effect of Cu addition on transformation temperature for annealed alloys.

The *M*_s_ temperature was raised by 9 °C from 137 °C to 146 °C when 3% Cu was used in place of Ni in the 0Cu alloy. Furthermore, the thermal hysteresis was reduced by 1 °C, from 23 °C to 22 °C, which is notable. These empirical results demonstrate the important effect of substituting 3% Ni for Cu, leading to higher transformation temperatures and less thermal hysteresis (Fig. 13).

**Fig. 13:** Effect of Cu addition on thermal hysteresis in case of solution treatment, aging and annealing.

For the 5Cu alloy, the *M*_s_ temperature increased by 10 °C from 137 °C to 147 °C while the *A*_f_ temperature of the 5Cu alloy increased by 9 °C to move from 163 °C to 172 °C as compared to the 0Cu alloy. In addition, it was noted that the thermal hysteresis dropped from 23 °C to 22 °C by 1 °C. These experimental results support the hypothesis that adding 5% Cu instead of Ni resulted in a notable increase in transformation temperatures and a slight decrease in thermal hysteresis.

The *M*_s_ temperatures of the 7.5Cu alloy were also increased as compare to 0Cu alloy, rising by 11 °C from 137 °C to 148 °C. The *A*_f_ temperature, which increased by 10 °C which ranged from 163 °C to 173 °C. In addition, it was observed that the thermal hysteresis dropped from 23 °C to 21 °C by 2 °C. These experimental findings led to the conclusion that replacing 7.5% Ni with Cu resulted in a large increase in transformation temperatures and a minor reduction in thermal hysteresis.

In a similar manner, the transformation temperatures of the 10Cu alloy were also increased as compared to the 0Cu alloy. The 10Cu alloy's *M*_s_ temperature rose by 16 °C, from 137 °C to 153 °C, while *A*_f_ temperature rose by 16 °C, from 163 °C to 179 °C. It was also observed that the thermal hysteresis dropped from 23 °C to 19 °C, a 4 °C drop. Based on these experimental findings, it was deduced that 10% Cu was substituted for Ni, which resulted in a large increase in transition temperatures and a modest reduction in thermal hysteresis.

Based on the aforementioned experimental data, it has been conclusively proven that the substitution of 10% Cu for Ni causes a considerable jump in transformation temperatures as well as a slight decrease in thermal hysteresis.

## Conclusions

The precipitation behaviour of an annealed TiNiPdCu alloy was carefully scrutinised as part of this work. This study's main goal was to thoroughly analyse and comprehend the variables that affect precipitation behaviour in order to show how they may be used to improve the dimensional stability of TiNiPd-based high-temperature shape memory alloys. Notably, the research found that micro-scaled TiPdCu and Ti_2_Pd precipitates were remarkably stable up to 500 °C.

Hard precipitates have historically presented difficulties when used to improve the characteristics of HTSMAs because of their propensity to negatively impact workability at room temperature. The alloy system and precipitation mechanism suggested in this paper, however, offer a fresh viewpoint. In order to take advantage of their optimum workability, this study suggests processing TiNiPd-based high-temperature shape memory alloys in a solution-treated form at ambient temperature. The final qualities of the alloy can then be customised by modifying the relevant process parameters. In summary, this novel method to precipitation provides a simple, quick process, especially from an industrial and practical perspective. It can now be used to increase the high-temperature operating range of TiNiPd-based alloys to above 500 °C. Beyond their homologous temperatures, where concerns about creep deformation could possibly weaken their functional qualities, this breakthrough is particularly relevant. The following are the main conclusions from this investigation:

1. A spinodal-type decomposition process within the TiNiPdCu alloy resulted in the development of two different types of precipitates (T_i2_Pd and TiPdCu).

2. When Cu was added in TiNiPd alloys, the density of the second phase precipitates is reduced and grain size increased.

3. At low and intermediate aging temperatures, two types of second phase precipitates (Ti_2_Pd, TiPdCu) were also detected. Resultantly the volume of martensite phase was reduced. However, at higher aging temperatures, the formation of those precipitates again disappeared and only the martensite phase was present.

4. It was obtained from DSC analysis that with the addition of Cu, transformation temperature increases and thermal hysteresis decreases significantly, which is suitable for high temperature applications *i.e.* high temperature sensors and actuators.

## Author contributions

Abid Hussain: conceptualization, validation, investigation, writing original draft, visualization; Afzal Khan: supervision, discussion, review & editing; M. Imran Khan: Co-supervision, review & editing, data analysis; Saif ur Rehman: project administration, discussion.

## Conflicts of interest

There are no conflicts to declare.

## Supplementary Material
